The article "Expression of GMFB in High-Grade Cervical Intraepithelial Neoplasia and Its Role in Cervical Cancer" was retracted in 2023. Reasons: signs of a paper mill; compromised peer review; unreliable results or conclusions.

# Expression of GMFB in High-Grade Cervical Intraepithelial Neoplasia and Its Role in Cervical Cancer

**DOI:** 10.1155/2022/7784921

**Published:** 2022-09-22

**Authors:** Jun Tian, Jianqing Wang, Yinxiu Chi, Zhongbao Han, Dongliang Zhang, Hu Zhang

**Affiliations:** ^1^Jiangsu Vocational College of Medicine, Yancheng, Jiangsu 222005, China; ^2^Department of Gynecology, Yancheng First People's Hospital, Yancheng, Jiangsu 222005, China

## Abstract

Cervical intraepithelial neoplasia (CIN) is a collective term for specific precancerous lesions associated with cervical cancer (CC). Although it has been affirmed with slow development of several levels of cellular changes, the existing poor prognosis calls for an urgent need to diagnose CIN at early stage and be aware of markers related to its pathogenesis and prognosis. We explored the expression level of a newly marker GMFB and its regulatory effect on CIN and CC. Patient samples and cell models were included. Bioinformatic studies were taken to predict its binding to miR-143-3p, miR-26b-5p, miR-191-5p, and miR-223-3p. Luciferase reporter and RNA pull-down assays were used to validate the prediction. Edu assay and flow cytometry were used to measure the regulation of GMFB on proliferation and apoptosis of CC cells. qRT-PCR was used for mRNA expression level detection. The results showed that GMFB was targeted by miR-143-3p, miR-26b-5p, miR-191-5p, and miR-223-3p. It had elevated expression in both CIN and CC samples. GMFB had highly prognostic value for CIN, and lymph node metastasis of CC was much associated with high GMFB expression level. Besides, silencing of GMFB inhibited CC cell proliferation and elevated cell apoptosis. In conclusion, we determined that GMFB has regulatory effect on high grade CIN and CC, which could lighten a novel way in exploring their pathogenesis and improving accuracy of prognosis.

## 1. Introduction

Cervical intraepithelial neoplasia (CIN) is a collective term for specific precancerous lesions associated with cervical invasive carcinoma [1]. CIN consists of cervical carcinoma in situ and cervical dysplasia and reflects the continuous progress of cervical cancer (CC). CC is a series of pathological changes, from cervical dysplasia (mild to medium severe) to carcinoma in situ, then early invasive carcinoma, and finally invasive carcinoma [2]. CIN is usually caused by certain types of human papillomavirus (HPV) and is subclassed into CIN 1, 2, and 3 as severity increases. It is diagnosed in view of the proportion of abnormal cells occupying the cervical epithelium [3]. CIN is classified as precancerous disease, even though only 9% of CIN 1 would develop into CIN 3 [4], and approximately 30% of CIN 3 would develop into CC [5].

The article "Expression of GMFB in High-Grade Cervical Intraepithelial Neoplasia and Its Role in Cervical Cancer" was retracted in 2023. Reasons: signs of a paper mill; compromised peer review; unreliable results or conclusions.

CC is the most common gynecologic malignancy, with the highest incidence rate of carcinoma in situ among patients aged 30 to 35 years, and that of invasive carcinoma among patients aged 45 to 55 years. In recent years, its onset population is becoming younger [6]. Researchers have found that persistent HPV infection, approximately 10–25 years, would induce CIN to progress into CC [7, 8]. These slow cellular changes calls for an urgent need to diagnose CIN at early stage and be aware of markers related to its pathogenesis and prognosis.

In 2020, LCoR expression was found to be correlated with CIN II progression, and RIP140 expression increases significantly as CIN grade progresses, underlining their potential role in the development of precancerous lesions [9]. In 2021, it was found in CIN samples that WAPL activates estrogen receptor signaling in early tumorigenesis of CIN, serving as a direct role in its induction [10]. Glia maturation factor-*β* (GMFB) is identified as the growth and differentiation factor of glia and neurons. It has been reported that GMFB induces ferroptosis in early diabetic retinopathy [11]. Besides, Sun et al. have pointed that GMFB is a novel biomarker and therapeutic target for hepatocellular carcinoma [12]. Nevertheless, there is few reports analyzing the role GMFB in high grade CIN or CC.

MicroRNAs (miRNAs) are small noncoding RNA molecules that combine with the 3′-untranslated region (UTR) of target mRNAs and modulate the expression of genes [13]. miRNAs affect the progression of several cancer types, including CC, by altering the biological activities of pro-or suppressor genes [14]. For example, miR-186-3p reduces tumorigenesis of CC by targeting IGF1 [15]. miR-411 hinders CC progression via binding to STAT3 [16]. In 2020, as miRNAs evolved into a versatile tool to distinguish genetical differences of cellular product [17, 18] and a diagnostic marker for various types of cancer, Wittenborn et al. discovered that a subpanel of six miRNAs (hsa-miR-26b-5p, hsa-miR-142-3p, hsa-miR-143-3p, hsa-miR-191-5p, hsa-miR-223-3p, and has-miR-338-3p) marked the CIN progress process and early stages of cervical squamous cell carcinoma [19]. Therefore, we set about investigation from the common target gene of these 6 miRNA markers and found that GMFB was targeted by miR-143-3p, miR-26b-5p, miR-191-5p, and miR-223-3p in common.

In summary, we proposed the hypothesis that GMFB has regulatory effect on high grade CIN and CC, which could lighten a novel way in exploring their pathogenesis and improving accuracy of prognosis.

## 2. Materials and Methods

### 2.1. Bioinformatic Studies

GMFB was found to be potentially targeted by miR-143-3p, miR-26b-5p, miR-191-5p, and miR-223-3p in common using the microRNA Target Prediction Database (miRDB, https://www.mirdb.org/), which is a dedicated database released in Dec 2018, included more than 8,500 experimental supporting articles on miRNA-target interactions. The overall survival curve with low/high GMFB TPM was referred from the Gene Expression Profiling Interactive Analysis (GEPIA, http://gepia.cancer-pku.cn/), which was developed by Professor Zhang Zemin Laboratory in 2017, Peking University. The platform includes RNA sequencing data of 8587 normal tissues and 9736 tumor tissues from The Cancer Genome Atlas (TCGA) and Genotype-Tissue Expression (GTEx) databases, mainly used for gene correlation analysis, dimensionality reduction analysis, gene expression analysis, survival analysis, similar gene prediction, etc.

The article "Expression of GMFB in High-Grade Cervical Intraepithelial Neoplasia and Its Role in Cervical Cancer" was retracted in 2023. Reasons: signs of a paper mill; compromised peer review; unreliable results or conclusions.

### 2.2. Patient Samples

A total of 15 cervical mucosal samples were collected from CIN patients during cervical biopsies, with 15 control samples collected from normal volunteers. A total of 15 carcinoma samples were collected from CC patients during hysterectomies, with another 15 control samples collected from normal volunteers. All patients were enroll in Yancheng First People's Hospital from Jan. 2020 to Jan. 2021 and informed with consent, along with normal volunteers. Patients with recurrence of cervical malignancies, undergoing treatment, or vaccination against HPV were excluded. This study was approved by the Ethics Committee of Yancheng First People's Hospital.

### 2.3. Cell Culture

H8 (BFN607200572, BLUEFBIO, Shanghai, China) cells were cultured in DMEM high glucose medium (Gibco, USA) supplemented with 10% fetal bovine serum (FBS) and 1% penicillin/streptomycin (P/S). C33A (CL-0045, Procell, Wuhan, Hubei, China) cells were cultured in Minimum Essential Medium (Gibco, USA) supplemented with 10% FBS+1% P/S. HEK293T (CL-0005, Procell, Wuhan, Hubei, China) cells were cultured in DMEM high glucose medium (Gibco, USA) supplemented with 10% fetal bovine serum (FBS) and 1% penicillin/streptomycin (P/S). All cells were grown at 95% air and 5% CO_2_ at 37°C and used 48 h later for subsequent experiments.

### 2.4. Cell Transfections

Short hairpin RNA (shRNA) against GMFB (sh-GMFB#1 and #2) and its negative control (sh-NC) were purchased from Fenghui Biotechnology (Changsha, Hunan, China). NC mimics, miR-143-3p mimics, miR-26b-5p mimics, miR-191-5p mimics, and miR-223-3p mimics were obtained from GenePharma Co., Ltd. (Shanghai, China). All plasmids were cotransfected into C33A cells using Lipofectamine™ 3000 transfection reagent (L3000015, Thermo Fisher, USA) according to the product's instructions. The cells were cultured at 37°C for 24 days and analyzed.

The article "Expression of GMFB in High-Grade Cervical Intraepithelial Neoplasia and Its Role in Cervical Cancer" was retracted in 2023. Reasons: signs of a paper mill; compromised peer review; unreliable results or conclusions.

### 2.5. Quantitative Real-Time Polymerase Chain Reaction (qRT-PCR)

Total RNA was extracted from C33A cells, cervical mucosal samples or carcinoma samples using TRIzol Reagent (15596-026, Ambion, USA). Hifair® II 1st Strand cDNA Synthesis Kit (11119ES60, Yeasen, Shanghai, China) was used for reverse transcription. SYBR Green FAST Mastermix was used for PCR process (Qiagen, Dusseldorf, Germany). The relative expression level was analyzed by the 2^−ΔΔCT^ method. GAPDH was used to normalize the expression of corresponding gene. The primer sequences were listed below: GMFB: (F) 5′-GTCCTGTTGGATGTAAGCCT-3′, (R) 5′-TGGTTAGTTCAGCTGTCTGG-3′; GAPDH: (F) 5′-TCAAGATCATCAGCAATGCC-3′, (R) 5′-CGATACCAAAGTTGTCATGGA-3′.

### 2.6. RNA Pull-Down Assay

RNA pull-down assay was conducted using CIN tissues and Pierce™ Magnetic RNA-Protein Pull-Down Kit (20164, Thermo Fisher, USA). Biotin-labeled probes targeting GMFB (bio-GMFB) and the negative control-biotin (bio-NC) were mixed with streptavidin magnetic beads (80 *μ*l), washed twice using TRIS buffer and incubated at room temperature for 25 min. The CIN tissues were lysed and mixed with pretreated magnetic beads labeled with probes overnight at 4°C. The magnetic beads were treated with 60 *μ*l elution buffer for 45 min at 37°C to extract GMFB -associated miRNAs, followed by qRT-PCR analysis.

### 2.7. Luciferase Reporter Assay

GMFB 3′UTR was loaded in pmirGLO dual-luciferase vectors (Promega, Madison, WI, USA). HEK293T cells cotransfected with NC mimics, miR-143-3p mimics, miR-26b-5p mimics, miR-191-5p mimics, and miR-223-3p mimics together with luciferase reporter vectors were seeded in 24-well plates. Luciferase activities were determined and normalized using Dual-Luciferase Reporter Assay System (Promega).

### 2.8. Edu Assay

Edu assay was conducted using EdU Cell Proliferation Kit (E607204-0050, Sangon Biotech, Shanghai, China). The EdU solution was added to the cell complete medium at 1 : 500 ratio to make 2x EdU medium and added to the original cell medium to obtain 1x EdU solution (the final concentration of EdU was 10 *μ*M). The 24-well plates were incubated with 300 *μ*l of EdU medium per well for 2 h and the medium was discarded. The plates were washed twice using 1X PBS for 5 min each. The plates were treated with 150 *μ*l of 4% paraformaldehyde per well at room temperature for 30 min, and then 100 *μ*l of the configured detection mixture per well free of light at room temperature for 30 minutes. The plates were washed with 300 *μ*l of 0.5% Triton X-100 cell permeabilization solution for 2 to 3 times for 10 min each and then added and treated with 300 *μ*l 1x Hoechst of staining solution per well for 20 to 30 minutes at room temperature. Cells were washed twice with 300 *μ*l PBS per well. A fluorescence microscope photograph was taken immediately after the staining.

The article "Expression of GMFB in High-Grade Cervical Intraepithelial Neoplasia and Its Role in Cervical Cancer" was retracted in 2023. Reasons: signs of a paper mill; compromised peer review; unreliable results or conclusions.

### 2.9. Flow Cytometry

Cells were centrifuged at 300 g and 4°C for 5 min. Afterwards, they were washed twice with precooled PBS, with a centrifugation at 300 g and 4°C for 5 min each time. Then, the cells were resuspended with 100 l 1 × binding buffer. Five *μ*l annexin V-FITC and 10 *μ*l PI Staining Solution were mixed with the cells. The reaction lasted for 10-15 min without light at room temperature. The mixture was treated with 400 L 1 × binding buffer and placed on ice, and the samples were detected by flow cytometry within 1 hour. The assay was conducted using annexin V-FITC/PI Apoptosis Detection Kit (A211-01, Vazyme, Nanjing, Jiangsu, China). FITC+ and PI− cells were defined as apoptotic cells.

### 2.10. Statistical Analysis

SPSS 20.0 statistical software was used for statistical analysis. All experiments were performed thrice independently. All the data were expressed as mean ± SD with *P* < 0.05 as a statistical significance. One-way analysis of variance (ANOVA) with Dunnett's test and student's *t*-test were used for comparison between groups. Sensitivity and specificity were calculated, with ROC curves built by mapping true-positive rate (sensitivity) against false-positive rate (1 − specificity).

## 3. Results

### 3.1. GMFB Is the Target of miR-143-3p, miR-26b-5p, miR-191-5p, and miR-223-3p

Previous paper [19] has discovered that miR-143-3p, miR-26b-5p, miR-191-5p, and miR-223-3p could serve as the biomarkers of CIN. miRDB was used to predict their common target, and it turned out that GMFB was targeted by these miRNAs in common (Figure 1(a)). Their binding sites were shown in Figure 1(b). Detected by RNA pull-down assay, bio-GMFB group had relatively higher enrichment of miR-143-3p, miR-26b-5p, miR-191-5p, and miR-223-3p in CIN tissue than bio-NC group (Figure 1(c)). Luciferase reporter assay results demonstrated that in HEK293T cells transfected with miRNA mimics, miR-143-3p, miR-26b-5p, miR-191-5p, and miR-223-3p groups, all showed relatively lower luciferase activity of pmirGLO-GMFB 3′UTR than cells transfected with NC mimics, suggesting that GMFB was directly targeted by miR-143-3p, miR-26b-5p, miR-191-5p, and miR-223-3p (Figure 1(d)). These results suggested that GMFB was the target of miR-143-3p, miR-26b-5p, miR-191-5p, and miR-223-3p.

### 3.2. GMFB Shows Upregulation in High-Grade CIN

Cervical mucosal samples were collected from normal volunteers and CIN patients to determine their GMFB expression levels. qRT-PCR results suggested that GMFB expression elevated significantly in CIN 2 and CIN 3 groups than in the control group, with evidently higher level in CIN 3 group than in the CIN 2 group (Figure 2(a)). Researches before have elucidated that the presence of HPV elevated the future risk of high grade CIN [20] and would even cause CC by a persistent infection [8]. Therefore, to further investigate GMFB expression in high-grade CIN, 15 patients with CIN 2-3 were divided into a positive group [10] and a negative group [5] according to HPV type, their information detailed in Table 1. Detected by qRT-PCR, HPV positive group showed significantly higher expression of GMFB than HPV negative group (Figure 2(b)). ROC curve analysis were performed using samples from 10 patients reported dead and 5 survived patients as negative control. The ROC curve was made according to the GMFB expression in corresponding samples, which showed that AUC was 0.9 (*P* = 0.0237 < 0.05), much close to 1, indicating GMFB had highly prognostic value for CIN (Figure 2(c)). These results showed that GMFB was upregulated in high-grade CIN samples, especially in HPV positive ones and could serve as the diagnostic marker for CIN prognosis.

The article "Expression of GMFB in High-Grade Cervical Intraepithelial Neoplasia and Its Role in Cervical Cancer" was retracted in 2023. Reasons: signs of a paper mill; compromised peer review; unreliable results or conclusions.

### 3.3. GMFB Is Upregulated in CC

To measure the expression level of GMFB in CC, paracancerous tissues and CC tissues were sampled as the control group and the cancer group. qRT-PCR results suggested that GMFB was significantly upregulated in the cancer group compared to that in the control group (Figure 3(a)). Overall survival curves provided by GEPIA database revealed that CC patients with low survival rate had high expression of GMFB, indicating that GMFB was related to the poor prognosis of CC (Figure 3(b)). To further determine the association between GMFB expression and the clinicopathological features of CC patients, 15 CC patients were enrolled for analysis with their information detailed in Table 2, which turned out that lymph node metastasis was much associated with high GMFB expression level (Figure 3(c)). Lymph node metastasis has been reported to be the main metastatic pathway and the most critical factor in the prognosis and recurrence of CC [21], thus confirming and explaining the poor prognostic value of GMFB in CC diagnosis. Detected by qRT-PCR, C33A cells showed significantly higher expression level of GMFB than H8 cells, again validating our finding, and was chosen to be our experimental subject in in vitro assays. These results suggested that GMFB was upregulated in CC tissues and cells and was related to the poor prognosis of CC.

### 3.4. GMFB Is an Oncogene in CC

To investigate the regulatory effect of GMFB on CC, sh-GMFB was transfected into C33A cells, interference efficiency detected by qRT-PCR (Figure 4(a)). Assessed by Edu assay, C33A cells transfected with sh-GMFB showed significantly less Edu positive cells (Figure 4(b)), indicating that sh-GMFB attenuated the proliferation of C33A cells. Furthermore, flow cytometry results suggested the apoptosis rate of C33A cells transfected with sh-GMFB was significantly increased (Figure 4(c)) compared to those transfected with sh-NC, demonstrating that sh-GMFB suppressed the proliferation of C33A by promoting apoptosis. These results suggested that GMFB was an oncogene in CC that regulate cell proliferation by controlling apoptosis.

The article "Expression of GMFB in High-Grade Cervical Intraepithelial Neoplasia and Its Role in Cervical Cancer" was retracted in 2023. Reasons: signs of a paper mill; compromised peer review; unreliable results or conclusions.

## 4. Discussion

CIN, serving as the precancerous lesions of CC, became the target direction for research related to CC in recent years. In 2013, Tornesello et al. mentioned that the detection of p16INK4a and Ki67 improves the identification of premalignant lesions that have a high risk to evolve into invasive CC, such as CIN [22]. In 2019, Huang et al. put forward that 54.8% of the gene mutations detected in CIN specimens occurred in CC specimens as well [23]. It was measured in [24] 2017 that the immunoreactivity of both cytoplasmic and nuclear p16INK4A was absent in normal cervical tissue, while positive in CIN 1 (25%), CIN 2 (50%), CIN 3 (75%), squamous cell carcinoma (75%), and adenocarcinoma (100%) suggesting the prognostic value of p16INK4A in the management of CC. These results were consistent with our finding that there exists specific proteins which were upregulated in both CC and CIN specimens. The qRT-PCR results suggested that GMFB expression was elevated significantly in the CIN groups than in the control group, with evidently higher level in the high-grade CIN group. The HPV positive group showed significantly higher expression of GMFB than the HPV negative group. The ROC curve analysis indicated that GMFB has highly prognostic value for CIN. CC specimen suggested that GMFB expression is elevated in CC tissues and cells and marked the poor prognosis of CC.

Glia maturation factor (GMF), first isolated from bovine brain in 1972, is a growth and differentiation factor [25], consisting of GMF-*γ* and GMFB. In 1989, GMFB was first purified from crude GMF [26]. Previous work has found that the expression of GMFB would elevate due to neuroinflammation and neurodegeneration, to modulate the expression of neurotrophin, granulocyte-macrophage colony-stimulating factor and superoxide dismutase [27]. In 2010, GMFB expression in serous ovarian carcinoma was found to be significantly enhanced than that in normal epithelium, benign serous adenoma, and borderline serous adenoma tissues and was associated with poor disease-free survival and overall survival [28]. In 2020, Sun et al. have proposed that GMFB expression was significantly upregulated in patients with hepatocellular carcinoma and positively coexpressed with tumor node metastases stage and histopathological grade of hepatocellular carcinoma [12]. However, the regulatory effect of GMFB in CIN and CC has few relevant reports.

The article "Expression of GMFB in High-Grade Cervical Intraepithelial Neoplasia and Its Role in Cervical Cancer" was retracted in 2023. Reasons: signs of a paper mill; compromised peer review; unreliable results or conclusions.

It has been reported that silencing of GMFB hindered cell proliferation and migration in hepatocellular carcinoma [12]. Our results proved GMFB to share similar behavior in CIN/CC as in other carcinomas, which has not previously been reported. Especially, to investigate the regulatory effect of GMFB on CC, Edu assay and flow cytometry were performed. The results suggested that compared to the control group, the sh-GMFB group showed suppressed proliferation of C33A, suggesting that GMFB is an oncogene in CC that regulate cell proliferation by controlling apoptosis.

There are several limitations in our study. First, the in vivo experiments were not performed to verify the effect of GMFB on tumor growth and metastasis. Additionally, whether GMFB promoted CC cell proliferation via regulating signaling pathways was unclear. Therefore, further researches will be carried out to perfect our study.

In conclusion, the regulatory effect of GMFB on CIN and CC was detected in our research, with the inner mechanism explored on account of apoptosis and proliferation, which proved for the first time that GMFB could be considered as a prognostic predictor for CIN/CC patients.

## Figures and Tables

**Figure 1:** GMFB is targeted by miR-143-3p, miR-26b-5p, miR-191-5p, and miR-223-3p (a) miRNAs listed in previous paper [19] and their common target GMFB predicted by miRDB. (b) Binding sites between GMFB and corresponding miRNAs predicted by miRDB. (c) Relative enrichment of miRNAs in CIN tissue bind to bio-GMFB/NC, detected by RNA pull-down assay. (d) Relative luciferase activity of pmirGLO-GMFB 3′UTR in HEK293T cells transfected by corresponding miRNA mimics. ^∗∗^*P* < 0.01, ^∗∗∗^*P* < 0.001.

**Figure 2:** GMFB shows upregulation in high-grade CIN (a) Relative GMFB expression in control and high-grade CIN groups (CIN 2 and CIN 3), detected by qRT-PCR. (b) Relative GMFB expression in HPV negative and positive groups, sampled from high-grade CIN patients, detected by qRT-PCR. (c) ROC curve of GMFB expression in dead and survived patients. ^∗∗^*P* < 0.01, ^∗∗∗^*P* < 0.001.

**Figure 3:** GMFB shows upregulation in high-grade CC (a) Relative GMFB expression in control and cervical cancer groups, detected by qRT-PCR. (b) Overall survival curves of patients with high/low GMFB expression, referred from GEPIA. (c) Relative GMFB expression in H8 and C33A cells, detected by qRT-PCR. ^∗∗∗^*P* < 0.001.

The article "Expression of GMFB in High-Grade Cervical Intraepithelial Neoplasia and Its Role in Cervical Cancer" was retracted in 2023. Reasons: signs of a paper mill; compromised peer review; unreliable results or conclusions.

**Figure 4:** GMFB is an oncogene in CC. (a) Relative interference efficiency of C33A transfected with sh-GMFB. (b) Proliferation of C33A cells and percentage of Edu positive cells, assessed by Edu assay. (c) Apoptosis rate of C33A cells, assessed by flow cytometry. ^∗∗^*P* < 0.01, ^∗∗∗^*P* < 0.001.

**Table 1:** List of patients with CIN 2-3.

No.	CIN level	Age	HPV type
1	2	37	Negative
2	2	32	Positive
3	2	33	Positive
4	2	28	Negative
5	3	48	Negative
6	3	41	Positive
7	3	43	Positive
8	3	42	Positive
9	3	34	Positive
10	3	31	Negative
11	3	36	Negative
12	3	42	Positive
13	2	40	Positive
14	2	27	Positive
15	3	41	Positive

**Table 2:** Association of GMFB expression and the clinicopathological features of patients with cervical cancer.

Characteristics	GMFB expression			
	Patient	Low	High	*P*
	*n* = 15	*n* = 7	*n* = 8	
Age				
50	8	3	5	0.6193
≥50	7	4	3	
FIGO stage				
I	11	5	6	>0.9999
II	4	2	2	
Tumor diameter				
≤4 cm	12	6	6	>0.9999
4 cm	3	1	2	
Differentiation grade				
Middle + low	9	5	4	0.6084
High	6	2	4	
Lymph node metastasis				
Yes	7	0	7	0.0014^∗∗^
No	8	7	1	
Vasoinvasion				
Yes	4	2	2	>0.9999
No	11	5	6	

^∗∗^Significant *P* values (*P* < 0.01).

## Data Availability

The corresponding author is responsible to the data, and we will provide the original data if necessary.
